# Analysis of Stress Response and Analgesic Effect of Remazolam Combined with Etomidate in Painless Gastroenteroscopy

**DOI:** 10.1155/2022/4863682

**Published:** 2022-08-03

**Authors:** Guihua Liu, Ying Xiong

**Affiliations:** Department of Anesthesiology, The Second Affiliated Hospital of Dalian Medical University, Dalian 116027, China

## Abstract

In order to explore more ideal intravenous anesthesia drug in clinical practice, the analgesic effect of remazolam combined with etomidate in painless gastroenteroscopy and its effect on stress response is investigated. A total of 100 patients are selected for the gastric disease screening, and they are randomly divided into the single-drug group and composite group, with 50 cases in each group. Etomidate, mazzolone, and etomidate are used to anesthetize the patients, and then, the effects of different solutions on analgesia, sedation, and stress response are compared and analyzed, and the adverse reactions are improved. The etomidate and red horse azole shimron composite etomidate anesthesia were applied, and the comparative analysis of different solutions of analgesic, sedative effect, and response to stress is conducted. Then, the improvement of adverse reactions is analyzed. The experimental results demonstrate that remazolam combined with etomidate anesthesia can reduce the level of pain mediators and enhance the analgesia and sedation effect. Meanwhile, combined anesthesia can reduce the stress response and adverse reactions of patients and shorten the examination period effectively.

## 1. Introduction

The risk of gastrointestinal dysfunction and hypertension will increase with age [1]. In order to make an effective diagnosis of the stomach diseases as soon as possible, the frequency of clinical examination of gastrointestinal tract is also increased accordingly. Stomach diseases can be divided into gastric functional diseases and organic diseases. Functional diseases include functional dyspepsia and gastroesophageal reflux [2]. Gastrointestinal endoscopy can cause abnormal changes in hemodynamics and stress response, which seriously threatens the life safety of patients. Therefore, reasonable selection of anesthetic and sedative drugs with a strong sedative effect is helpful to alleviate the stress response and prognosis of patients undergoing gastrointestinal endoscopy. Etomidate is an anesthetic widely used in clinical practice. It has the advantages of fast response, short response time, and high safety. Its good anesthetic effect has been recognized [3]. It is soluble in chloroform, insoluble in acetone, and insoluble in ether. Its effect on the central nervous system is similar to that of barbiturates. Hypnosis is strong, and its efficacy is about 12 times than that of thiopental sodium, without the analgesic effect. Anesthesia takes effect quickly. Anesthesia occurs 20 seconds after intravenous injection. Anesthesia lasts for about 5 minutes and wakes up quickly [4]. Compared with thiopental sodium, the anesthesia intensity is higher, and the effect on respiratory and circulatory system is smaller. Intravenous anesthesia can increase coronary blood flow by 19% and reduce resistance by 19% [5]. In addition, it has little impact on the respiratory and circulatory system, with transient respiratory depression. It can slightly reduce systolic blood pressure and slightly increase heart rate. It can affect liver and kidney functions, reduce brain oxygen consumption, reduce cerebral blood flow, and intracranial pressure [6].

Remazolam is a new type of ultrashort acting benzodiazepine anesthetics, which has the characteristics of predictable sedation time and rapid recovery in painless gastroscopy [7]. Propofol is a commonly used intravenous anesthetic in clinical work, which has the advantages of rapid onset, short onset time, and rapid recovery. Propofol and midazolam can achieve certain effects in clinical anesthesia. However, patients have a higher risk of adverse cardiovascular and respiratory depression after anesthesia. Therefore, it is urgent to find more ideal intravenous anesthetics in clinical practice [8]. Remazolam is a new anesthetic with certain safety and sedative effect, and has been clinically recognized [9]. However, from a clinical point of view, the analgesic effect of remazolam combined with etomidate in painless gastroenteroscopy, and its effect on stress response should be investigated deeply and comprehensively.

The rest of this paper is organized as follows: Section 2 demonstrates the related work. Then, the methods of anesthesia and evaluation indicators are presented in Section 3.  Section 4 presents the results and analysis.  Section 5 concludes the paper and gives the future work.

## 2. Related Work

With the growth of age, people's gastrointestinal function decreases and poor eating habits increase the damage of gastrointestinal function [10]. This has caused the incidence rate of gastrointestinal diseases to increase year by year. In addition, with the gradual improvement of medical technology and the in-depth development of the concept of comfortable medical treatment, clinical painless colonoscopy has become a widely used and effective certification examination project [11]. It has important guiding significance for the examination of gastric diseases. It should be noted that different anesthetics will directly affect the anesthesia and examination results. Therefore, it is of great significance to actively select anesthetics with low stress response and high safety in painless colonoscopy [12].

Etomidate is a nonbarbiturate sedative with strong sedative effect and short duration. It is widely used in endoscopic anesthesia, and its sedative effect has been certified, but certain adverse reactions still exist [13]. Currently, propofol and midazolam are the most commonly used drugs in clinical anesthesia, but there are still some shortcomings. Remazolam is a new anesthetic drug improved on the basis of midazolam, which makes up for the poor sedation effect of midazolam in clinical anesthesia. Kim et al. [14] showed that remazolam can achieve sedative and analgesic effects similar to propofol. The sedation score, pain score, and pain mediators of patients in the combination group are significantly improved or decreased, which indicated that remazolam could enhance the sedation and analgesic effect. From the perspective of pharmacological characteristics to analyze its mechanism may be as one of the central nervous system drugs of benzodiazepine of azole shimron, can make the neurotransmitter passing through anesthesia nerve is blocked, decrease PGE2 and IL-17, secretion and expression of pain medium, and then make the pain medium effects on peripheral nerve endings to effectively alleviate pain, In addition, remazolam modified on the basis of midazolam adds methyl propionate side chain, which can directly act on *γ*-aminobutyric acid TYPE A receptor and exert certain sedative effect through this pathway [15].

Pain, trauma, and other factors will lead to the activation of prostaglandin intraoxidase reductase, and then trigger an inflammatory cascade, which activates the release of a large number of inflammatory factors, and then trigger the stress response [16]. Above study suggests that remazolam combined with etomidate can improve the stress response generated by gastroenteroscopy in patients. The mechanism is that remazolam can play an anti-inflammatory role and effectively reduce the level of inflammatory factors in patients after surgery. Thus, the inflammatory cascade reaction and stress response caused by excessive secretion of inflammatory factors can be effectively alleviated [17–19]. Research shows that the time of free breathing is shortened to a certain extent after patients wake up. This suggests that erythromazzolone can obtain a good sedative effect. In addition, it has no effects on human metabolites and organ functions and can minimize the negative impact of drug anesthesia on patients. The reason may be that remazolam can be rapidly metabolized by tissue esterase in the human body, and the metabolites generated are inactive. Therefore, sedation can subside rapidly, and the patient's breathing and consciousness can be restored in a short time [20, 21].

## 3. Methods of Anesthesia and Evaluation Indicators

### 3.1. General Information

A total of 100 patients who underwent gastroenteroscopy in our hospital from January 2021 to January 2022 are screened and randomly divided into single-drug group and compound group, with 50 patients in each group. In the single-drug group, the male/female ratio is 23/27, the age is 44∼63 years, and the average age is (53.61 ± 9.42) years. The ASA grade is I/II is 22/28. Besides, there are 15 cases of gastric cancer, 16 cases of chronic gastritis, and 19 cases of gastric ulcer. There are 13 cases of gastric cancer, 17 cases of chronic gastritis, and 20 cases of gastric ulcer in the compound group. There is no statistically significant difference in baseline data of all subjects after comparison (*P* > 0.05), which can be compared effectively. Inclusion criteria are as follows: patients who underwent colonoscopy in our hospital; patients with ASA grade I ∼ II; after clarifying the research content and significance, the informed consent is signed voluntarily; there are no obvious allergic reactions or contraindications to remazolam and etomidate used in this study. Exclusion criteria are as follows: combined diseases of cardiovascular, respiratory, and endocrine systems; complicated with vital organ failure; severe allergy to the drugs used in this study or long-term use of sedative drugs before participating in the study; there are mental diseases and cognitive disorders.

The study is approved by the medical ethics committee of the hospital. SPSS 21.0 software is used as a statistical analysis tool for the study data. ($\bar{x}\pm s$) is used to represent the normal measurement data, the *t* test is used, the count data are expressed as *n* (%), the *χ*^*2*^ test, and *P* < 0.05 is statistically significant.

### 3.2. Methods of Anesthesia

All patients need regular fasting for 12 hours and drinking for 8 hours before examination. Lateral prone position is taken, oxygen is inhaled by nasal catheter at 3.0 L/min, and ECG and heart rate are monitored by DASH4000 multifunctional monitor (GE). In the single-drug group, 0.9% normal saline is injected, and etomidate (Jiangsu Hengrui Pharmaceutical Co., Ltd., Production lot no. 20171015) is injected 2 min later at a rate of 0.2 mg/(kg/min). On the basis of the single-drug group, anesthesia induction is performed with remazolam (Jiangsu Hengrui Pharmaceutical Co., Ltd., Batch No. 200725) at 12 mg/(kg/h), and anesthesia is maintained at 1.0-2.0 mg/(kg·h). After the patient's consciousness disappeared, gastroenteroscopy (Olympus, Japan, model: CV-170) is performed. According to the patient's physical reaction during the examination, 4–6 mg etomidate is added appropriately. After the gastroenteroscopy reached the ileocecal area, the administration is stopped.

### 3.3. Evaluation Indicators

#### 3.3.1. Pain Mediators and Stress Indicators

5 ml fasting venous blood of the subjects is collected before and after surgery 12 h and deposited for 1 hour. After that, a low-speed centrifuge is used to centrifuge for 15 min with a centrifugal radius of 6.5 cm and rotation speed of 3500 r/min. The serum and plasma are separated and stored in a refrigerator at −4°C for examination. Enzyme-linked immuno sorbent assay (ELISA) is used to detect the levels of pain mediators, including prostaglandin (E2, PGE2) and interleukin-17 (IL-17) levels. Stress indicators included cortisol (Cor), adrenaline (*A*) and noradrenaline (NA) levels in peripheral venous blood. The two time points are marked *T*1∼*T*2.

### 3.4. Observation Indicators

The observation indicators include (1) the recovery time of spontaneous breathing and recovery time of each group are recorded and compared; (2) stress indexes and pain mediators at different time points in each group are recorded and compared; (3) visual analogue scale (VAS) score and Ramsay sedation score of each group are recorded and compared. The total VAS score is 0∼10 points, and patients drew lines on 10-scale white paper according to the pain degree. The pain degree increased with the increase of the score. The total score of Ramsay sedation score is 0∼6, 1∼3, and 4∼6 indicated that the patients are awake and asleep. The sedative effect decreased as the score increased; (4) adverse reactions such as nausea and vomiting, respiratory depression, dizziness and headache, and hypoxemia in each group are recorded and compared.

## 4. Results and Analysis

### 4.1. Anesthetic Indicators

Compared with the single-drug group, the compound group had shorter recovery time of spontaneous breathing and recovery time with statistical differences (*P* < 0.05), as shown in Table 1.

### 4.2. Changes of Stress Indexes and Pain Mediators at Different Time Points

Table 2 shows the stress index changes at different time points ($\bar{x}\pm s$, *n* = 50).  Figure 1 demonstrates the changes of stress indicators. In addition, the changes of pain mediators at different time points ($\bar{x}\pm s$, *n* = 50) are illustrated in Table 3, and the changes of pain mediators are shown in Figure 2. It can be observed that the levels of PGE2, IL-17, Cor, A, and NA at *T*2 in the single-drug group and the compound group are all higher than those at *T*1, and the levels of 5 indexes are lower in the compound group, with statistical differences (*P* < 0.05).

### 4.3. Comparison of Analgesic and Sedative Effects

The composite group had lower VAS score and higher Ramsay sedation score than the monotherapy group, both of which are statistically significant (*P* < 0.05), as shown in Table 4 and Figure 3.

### 4.4. Occurrence of Adverse Reactions

Table 5 is the proportion of adverse reactions (*n* = 50, %). It is clearly evident from Table 5 that the incidence of adverse reactions is significantly lower in the compound group than in the monotherapy group (*P* < 0.05).

## 5. Conclusions and Future Work

In this study, the analgesic effect of remazolam combined with etomidate in painless gastroenteroscopy and its effect on stress response is investigated. Painless stomach and the application of red mazzolone combined with etomidate anesthesia solution can help reduce patients' moderate pain and improve the clinical effect of analgesia and sedation. The combined anesthesia scheme can alleviate the stress reaction and adverse reaction of gastric examination and can make patients recover consciousness quickly, so as to effectively shorten the examination cycle. Remazolam combined with etomidate anesthesia is worthy of clinical promotion in painless gastroscopy.

Due to the small sample size and incomplete observation indicators, there is a room for further improvement in the research ideas. Therefore, in the follow-up study, we should increase the sample size and observation indicators to carry out large sample and multicenter in-depth research.

## Figures and Tables

**Figure 1:** Changes of stress indicators.

**Figure 2:** Changes of pain mediators.

**Figure 3:** Changes of analgesia and sedation scores.

**Table 1:** Indicators of anesthesia ($\bar{x}\pm s$, *n* = 50).

Group	Recovery time of spontaneous breathing (min)	Wake up time (min)
Single-drug group	8.64 ± 1.89	13.32 ± 3.43
Composite group	6.14 ± 1.78	9.24 ± 2.77
*t*	6.809	6.544
*P*	<0.001	<0.001

**Table 2:** Stress index changes at different time points ($\bar{x}\pm s$, *n* = 50).

Group	Cor (*μ*g/L)		A (*μ*g/L)		NA (*μ*g/L)	
	*T*1	*T*2	*T*1	*T*2	*T*1	*T*2
Single-drug group	223.34 ± 21.69	313.32 ± 25.43	81.34 ± 13.67	139.32 ± 21.23	343.24 ± 24.69	513.52 ± 29.43
Composite group	219.24 ± 21.58	277.34 ± 28.77	79.24 ± 14.78	117.23 ± 22.54	339.84 ± 25.21	447.24 ± 27.37
*t*	0.948	6.626	0.738	5.045	0.681	11.661
*P*	0.346	<0.001	0.463	<0.001	0.497	<0.001

**Table 3:** Changes of pain mediators at different time points ($\bar{x}\pm s$, *n* = 50).

Group	PGE2 (ng/L)		IL-17 (ng/L)	
	*T*1	*T*2	*T*1	*T*2
Single-drug group	98.62 ± 11.19	248.22 ± 17.23	4.82 ± 1.33	9.68 ± 1.43
Composite group	96.13 ± 10.98	166.21 ± 15.32	4.84 ± 1.29	7.52 ± 1.19
*t*	1.123	25.152	-0.009	8.210
*P*	0.264	<0.001	0.993	<0.001

**Table 4:** Analgesia and sedation scores ($\bar{x}\pm s$, *n* = 50).

Group	VAS score	Ramsay sedation score
Single-drug group	8.64 ± 1.89	1.42 ± 0.33
Composite group	6.14 ± 1.78	2.64 ± 0.77
*t*	6.809	−10.298
*P*	<0.001	<0.001

**Table 5:** Proportion of adverse reactions (*n* = 50, %).

Group	*N* and *V*	Respiratory depression	Dizziness headache	Hypoxemia	Total incidence
Single-drug group	2 (4.00)	3 (6.00)	2 (4.00)	3 (6.00)	10 (20.00)
Composite group	1 (2.00)	1 (2.00)	1 (2.00)	0 (0.00)	3 (6.00)
*χ * ^2^					4.332
*P*					0.037

## Data Availability

The data used to support the findings of this study are available from the corresponding author upon request.
